The article "Impact of Low-Carbon City Policy on Enterprise Investment Efficiency: Based on the Heterogeneity of Chinese Urban Culture" was published in 2022. Journal: J Environ Public Health.

# Impact of Low-Carbon City Policy on Enterprise Investment Efficiency: Based on the Heterogeneity of Chinese Urban Culture

**DOI:** 10.1155/2022/1998278

**Published:** 2022-09-22

**Authors:** Yishuai Shi, Yuhang Guan, Li Li

**Affiliations:** ^1^Business School, Nankai University, Tianjin 300110, China; ^2^School of Management, Yulin University, Yulin 719000, China

## Abstract

Based on panel data of Chinese listed companies, this paper estimates the impact of low-carbon city policy (LCCP) on enterprise investment efficiency (EIE) by the heterogeneous timing difference in differences (HTDID) method and examines the heterogeneous effect of urban culture on the impact. The results show that LCCP improves EIE, and the research conclusion passes the robustness tests. Mechanism analysis reveals that LCCP mainly acts on EIE along two paths: promoting enterprise technological innovation and easing financing constraint. But the LCCP does not have a significant effect on resource allocation. On urban culture heterogeneity, the ecological wisdoms of green urban culture and Confucian culture, such as benevolence to all beings and the harmony between man and nature, help to enhance the promoting effect of LCCP on EIE. From the perspectives of the synergistic development between formal and informal institutions and of urban cultural governance, this research provides important reference and data support to EIE improvement.

## 1. Introduction

Global warming, a consequence of greenhouse gas emissions, exposes human beings to multiple risks, including sluggish economic growth and worsening living environment. To address these risks, the National Development and Reform Commission of China issued the *Notice on Launching the Pilot Program of Low-Carbon Provinces and Low-Carbon Cities* in 2010, kicking off the piloting of low-carbon city development. In the meantime, the Chinese economy is moving from the high-speed growth stage to the high-quality development stage. The further decline of industrial production efficiency has severely bottlenecked the macroeconomic growth of China in recent years. The low-carbon city policy (LCCP) requires cities to clarify their development strategies, principles, and directions during the pursuit of low-carbon development; accelerate the research and development, promotion, and application of low-carbon technologies; build a low-carbon industrial system characterized by greenness, environmental friendliness, and high recyclability; and implement the industrial policies, fiscal and tax policies, and technology promotion policies for low-carbon development, aiming to strengthen the driving role of low-carbon technology innovation on economic development. Enterprises are the most important participant and contributor in the construction of low-carbon cities. Being major emitters of carbon dioxide, enterprises are the core organizers of low-carbon product research and development and need to improve investment efficiency, one of the most effective ways to reduce carbon emissions and lead the construction of low-carbon cities. In the context of China's economic transformation, culture lies at the core of the informal institution and significantly affects economic and social development. The implementation of the LCCP is inseparable from the cultural foundation at the city level. Therefore, it is particularly important to explore the impact of LCCP on enterprise investment efficiency (EIE) and consider the role of urban culture for the implementation of policies. Facing the realistic needs of ecological protection and high-quality development, this paper is aimed at answering the following questions: does China's LCCP help improve EIE? Under the influence of culture, an important informal institution, does the relationship between LCCP and EIE varies with the culture of specific cities?

Rich results have been drawn on the evaluation of the effect of LCCP. Many scholars used the data of Chinese listed companies to evaluate the impact of LCCP on the total factor productivity [1]. For example, Song et al. [2] measured the impact of LCCP on energy efficiency. Cheng et al. [3] discussed the effect of low-carbon city construction on green growth. Chinese scholars have also explored the relationship between LCCP and economic efficiency extensively. For instance, Z. Wang and H. Wang [4] found that the LCCP can significantly promote the high-quality development of enterprises, both in terms of the total factor productivity and sustainable development. Zhao et al. [5] and Guan et al. [6] proved the positive effect of LCCP on the total factor productivity of enterprises. Fan and Liu [7] discovered that the LCCP has significantly improved the total factor energy efficiency. The existing literature provides profound insights for the effect evaluation of LCCP. But there are some shortcomings. Firstly, the existing research on LCCP emphasizes environmental performance and economic performance, over the impact of LCCP on EIE. To enhance the development resilience and core competitiveness of enterprises, it is crucial to take low-carbon city piloting as a strategic opportunity to inject new vitality into the improvement of EIE, by boosting the enthusiasm and creativity of implementing the climate action vision. Therefore, it is important to explore the impact of LCCP on EIE, a weak link in the existing research. Secondly, the piloting effect of LCCP is closely associated with the urban culture, yet the factors of urban culture have not been thoroughly investigated. Thus, it is of great academic value to systematically evaluate the action and effect of China's LCCP on EIE and examine the effects of urban cultural factors.

Based on the above analysis, this paper intends to reveal the impact mechanism of LCCP on EIE and to empirically test that impact. Taking the LCCP as a quasinatural experiment, the authors estimated the impact of LCCP on EIE, using the heterogeneous timing difference in differences (HTDID) method, and alleviate the endogenous bias through a series of robustness tests. In addition, urban green culture and Confucian culture were taken as examples; the heterogeneous impact of urban culture was examined, revealing the key role of cultural governance in the implementation of LCCP. This is another defining feature of this research. The research findings help to examine the achievements of low-carbon city construction, deepen the understanding of the factors affecting EIE, and provide reliable suggestions for promoting high-quality economic development while implementing low-carbon governance.

The main contributions are as follows: firstly, scholars have not reached a consensus on how environmental regulation affects economic efficiency of enterprises [8–11]. At the same time, the existing literature only focuses on the overall impact of environmental regulation intensity on EIE, without going to the details. This paper examines the implementation effect of LCCP from the perspective of investment efficiency and expands the research framework for scientifically quantifying the implementation effect of the policy on the basis of overcoming self-selection of samples, thereby alleviating endogeneity and eliminating other policy interference. Secondly, the mechanism of LCCP on EIE is verified; that is, LCCP will affect EIE through technological innovation effect and alleviating financing constraint effect, and LCCP does not produce resource allocation effect. Thirdly, the analysis on urban culture heterogeneity discovers that both urban green culture and Confucian culture offer a favorable environment for the orderly promotion of LCCP.

## 2. Theoretical Analysis and Hypotheses

### 2.1. LCCP and EIE

Under the global trend of carbon reduction, China launched the first batch of low-carbon pilot projects in 2010. Each pilot region was required to explore a low-carbon development model according to its own conditions. Subsequently, the second and third batches of pilot projects were determined in 2012 and 2017, respectively. The pilot regions need to complete the following tasks: establishing a responsibility system for carbon control target, setting up a carbon emission data statistics and management system, formulating supporting policies for low-carbon development, constructing a low-carbon industrial system, and advocating the low-carbon green lifestyle. This paper intends to demonstrate the impact of LCCP on EIE from three aspects: technological innovation effect, financing constraint effect, and resource allocation effect.

Specifically, the technological innovation effect refers to the influence of LCCP over EIE via technological innovation. LCCP is an environmental regulation policy proposed by China at the city level to reduce carbon emissions [12]. The influence of LCCP over enterprise technological innovation is mainly theorized based on the Porter's hypothesis, which holds that environmental regulation has two impacts on enterprise decision-making: (1) environmental regulation will push up the production cost of enterprises and squeeze their profit margin, forcing them to cut research and development (R&D) expenditure and increase financial investment. In this way, environmental regulation will eventually suppress EIE. (2) Environmental regulation stimulates enterprises to invest more on R&D [13, 14], forcing them to improve profitability by upgrading equipment or investing in relevant technologies. These means help to offset the extra expenditure brought by environmental regulation [15, 16]. In this case, the enterprises will become more efficient in production and investment [17, 18]. In addition, Porter's hypothesis believes that environmental regulation can manifest as an external pressure, which encourages enterprises to overcome investment inertia and complements with the internal governance mechanism, exerting an incentive effect on EIE [19]. The key areas of low-carbon city construction are industry, construction, transportation, energy supply, and waste management. Therefore, LCCP mainly guides these industries to achieve low-carbon development, so as to control greenhouse gas emissions at the city level. In this process, enterprises are guided to implement technology research and development, in order to make energy use more efficient. In addition, the central government treats local pilot programs seriously. Being selected as a piloting site is both an honor and a responsibility. Thus, local government is enthusiastic about environmental governance, once the region is selected for the piloting of low-carbon cities. Enterprises are encouraged to improve technology to achieve green and low-carbon development, which in turn enhances enterprise technological innovation and thus improves EIE. There are different views on the features of China's LCCP. Some hold that the LCCP is China provides weak incentives, and some argue that it exists as weak constraints. The pilot capacity-building projects only receive a small amount of financial support. The local governments do not receive additional financial and policy resources from the competent national authorities. Neither do they face assessment pressure like performance evaluation and project review. As a result, some pilot work fails to achieve the desired results. Therefore, it is difficult to improve EIE by promoting technological innovation. The above analysis shows the needs to verify the technological innovation effect of LCCP on EIE.

The financing constraint effect refers to the influence of LCCP over EIE via easing the financing constraint. To integrate the concept of low-carbon development into the production and operation of enterprises, the government has continuously stepped up its support for enterprises. Local governments have made bold explorations and attempts with the help of the autonomy granted by their superiors, such as tax relief, financial subsidies, loan discounts, special funds, and talent incentives, aiming to help enterprises to expand financing channels. Banks and other financial institutions regard the government support and subsidies as implicit guarantees and lower the credit threshold for the enterprises receiving such support and subsidies. For example, the low-carbon urban plans of the pilot regions all cover various financial policies, namely, the special funds for low-carbon development, subsidies for specific industries, preferential loan interest rates, and tax reductions and exemptions. Through capital allocation, these financial policies guide enterprises to reduce investment in polluting projects and invest more funds in green industries and environment-friendly production processes [20], thereby alleviating the financing constraint and enhancing EIE.

The resource allocation effect refers to the influence of LCCP on EIE by affecting enterprise resource allocation. On the one hand, the implementation of LCCP, whether it is the formulation of emission reduction requirements, the collection of pollution taxes, or the trading of pollution rights, will generate new costs, which will cause enterprise production to deviate from the original optimal state. The reason is that environmental regulation will increase the corporate cost of pollution control and system compliance [21]. Some enterprises may reduce production activities and even shut down the production facilities [22, 23]. In other words, environmental regulation will disrupt the normal investment of enterprises and reduce investment efficiency. On the other hand, the theory of bounded rationality says that low-carbon city piloting can strengthen the awareness of resource allocation efficiency among enterprises, pointing out the possible direction for improving that efficiency. Under the constraints of the low-carbon city pilot policy, the carbon reduction cost of enterprises with high emissions and low production efficiency may approach or even exceed their normal operating income. At this time, the enterprises face multiple pressures, such as relocation, merge, transfer, shutdown, or withdrawal, in order to utilize resources more efficiently. In the light of long-term economic benefits, a rational enterprise will choose to improve the efficiency of resource allocation and thus reduce or eliminate the pressure from environmental costs. Meanwhile, low-carbon city piloting provides preferential policies and fund supports to enterprises in various forms. Enterprises can seize the opportunities and utilize the favorable conditions to optimize the internal organizational structure, improve coordination and cooperation, and enhance the ability to identify investment opportunities, thereby improving EIE.

Through the above analysis, the following hypotheses were presented.

**Hypothesis 1 .**

LCCP can promote EIE.

**Hypothesis 2 .**

LCCP can suppress EIE.

**Hypothesis 3 .**

LCCP influences EIE via technological innovation effect.

**Hypothesis 4 .**

LCCP influences EIE via financing constraint effect.

**Hypothesis 5 .**

LCCP influences EIE via resource allocation effect.

### 2.2. Heterogeneity of Urban Culture

Urban culture is mainly defined in two ways: deducing from the definition of culture and defining by the features of the city itself. Concerning the first way, urban culture is defined as the sum of material and spiritual wealth created by people in the city and is the overall form of their living conditions, behavior patterns, spiritual characteristics, and urban features. Concerning the second way, urban culture is defined as a cultural model with urban characteristics jointly created by citizens in the long-term life process and is the sum of urban living environment, lifestyle, and living habits, according to the *Chinese and Foreign Urban Knowledge Dictionary*. It is a rather complex and diversified issue. Urban culture, as a way of communication between people and cities, is rooted in the soil of urban historical development and is the characteristic gene of a city. Urban culture has strong regional characteristics, and its development is largely affected by administrative division. Therefore, different cities may vary significantly in terms of culture. As an informal system, culture has an important impact on the economy and enterprise behavior. Urban green development is impossible without the support and guidance of culture. The promotion and implementation of LCCP cannot be detached from the special “soil” of urban culture, especially the green gene in culture. Urban green culture is the value and philosophy of ecoenvironment protection and resource utilization with urban characteristics, both of which gradually form in the process of urban operation and management. As the main body of Chinese traditional culture, Confucian culture has a subtle influence on the behavior of Chinese people. Its ecological ethics and wisdom are highly consistent with modern concepts like ecological civilization and green development. Both urban green culture and Confucian culture carry the gene of green culture, exerting an important impact on the implementation of LCCP. Therefore, this paper takes urban green culture and Confucian culture as examples to explore the different roles of urban culture differences in the implementation of LCCP.

Confucian culture has a long history of development. After more than two thousand years, Confucian culture has gradually established the core values and moral norms of Chinese culture and has become the ethics of “daily use without knowing.” With a low per capital ecological wealth, China faces a growing mismatch between the public's pursuit of high-quality life and the insufficient supply of urban development resources. *The Outline of the Tenth Five Year Plan for National Economic and Social Development* proposed to break the extensive “black” development model with GDP growth as the fundamental goal, switching to a resource-saving, environment-friendly, and green path towards sustainable development. Since then, urban green culture has been gradually formed through urban green operation and management and imperceptibly affected the public's values and decision-making. Therefore, Confucian culture and urban green culture are the representatives of traditional culture and emerging culture, respectively, and carry the very gene of green culture. Meanwhile, the two cultures vary greatly from city to city.

Urban green culture refers to the values and philosophy of ecoenvironmental protection and resource utilization with urban features. These values and philosophy are formed gradually during urban operation and management. Firstly, urban green culture can promote enterprises to generate cohesive and centripetal forces, which are friendly to the environment. By giving play to the guiding role of culture, the awareness of environmental protection can be formed subtly, and employees are encouraged and instructed to care for the environment and make concerted efforts for environmental protection. Secondly, urban green culture will form a binding force in enterprises through institutional norms and responsibility requirements. The social and environmental responsibilities that enterprises should undertake in production and operation will be stressed, motivating enterprises to develop the relevant institutions. Hence, urban green culture will lay a good basis for the promotion and implementation of LCCP and actively shape the influence of LCCP over EIE.

The behavior of enterprises is affected by the institutional environment [24]. China is currently going through a period of economic transformation. The formal institution in the country is not yet perfect, giving informal institution an important position. Culture, the core of the informal institution, significantly affects economic and social development. Here, Confucian culture is included in the research framework of the impact of LCCP on EIE, mainly for two considerations: firstly, Confucian culture is the merit of Chinese traditional culture, which has imperceptibly influenced the people's behavior for thousands of years [25], and shapes the values and business philosophy of Chinese entrepreneurs [26]. It is unsurprising that the business decisions of enterprises are, to a certain extent, affected by Confucian culture. In addition, China has been actively promoting its traditional culture in recent years, which deepens the influence of Confucian culture in the contemporary era. Secondly, Confucianism embodies rich ecological ethics. The modern concepts of ecological civilization and green development are highly consistent with the Confucian ideas of “harmony between man and nature” and “benevolence for all things.” The ecological wisdom advocated in Confucian culture cultivates the green development awareness among enterprises and drives the green transformation from the inside. The Confucian concepts of righteousness and profit guide enterprises to sacrifice interest for righteousness, actively undertake social responsibilities, and move away from the extensive growth model of the economy. The ideas of prudence and introspection make enterprises more aware of environmental self-discipline, forming an internal self-supervision mechanism, and promote them to actively practice the development of low-carbon cities. Therefore, Confucian culture will play a role in the influence of LCCP over EIE.

To sum up, the following hypotheses were presented.

**Hypothesis 6 .**

The stronger the urban green culture, the more LCCP improves EIE.

**Hypothesis 7 .**

The stronger the Confucian culture, the more LCCP improves EIE.

## 3. Empirical Design

### 3.1. Identification Strategy

Taking the low-carbon city piloting policy of China as an example, this paper explores how LCCP affects EIE. Since the piloting program starts from different years in different cities, the HDID method was adopted to recognize the influence of LCCP over EIE. The benchmark econometric model can be designed as

(1) $$\begin{array}{c} I\text{n}{vesteff}_{i,t+1}=\alpha +\beta {LCC}_{i,t}+{X_{i,t}}^{\prime }\gamma +\mu_{i}+\sum Y\text{ear}+\sum I\text{ndustry}+\sum P\text{rovince}+\varepsilon_{i,t}, \end{array}$$

where *i* and *t* are the serial numbers of enterprises and years, respectively; Investeff_*i*,*t*+1_ is EIE; LCC_*i*,*t*_ is the low-carbon piloting state of the registered city of the enterprise; *X*_*i*,*t*_ is a series of control variables; *μ*_*i*_, ∑Year, ∑Industry, and ∑Province are the fixed effects of individuals, years, industries, and provinces, respectively; *ε*_*i*,*t*_ is a random error; and *β* is the estimate of HDID, the key index of this research.

### 3.2. Samples and Data Sources

The research samples are the nonfinancial Chinese enterprises listed in the A-share board of Shanghai and Shenzhen stock exchanges from 2007 to 2016. Financial enterprises were excluded from the samples, mainly for the following two reasons: firstly, the financial industry, especially the banking industry, is more special than general industries. For example, many banks earn profits from off-balance sheet businesses. Bias is unavoidable if listed banks are analyzed based on the three major financial statements. Secondly, the financial enterprises have different financial statement requirements different from nonfinancial enterprises, because of the difference in business model between the financial industry and other industries. The statement structure and main accounting items of the financial industry are also different from those of general industries. The following samples were also excluded: the samples receiving special treatment (ST) or facing delisting risk (∗ST), the enterprises issuing both A-shares and B-shares, and the enterprises with key variables missing. The relevant data were collected from China Stock Market & Accounting Research (CSMAR) database and WIND database.

### 3.3. Important Variables and Measurements

#### 3.3.1. Measurement of Low-Carbon City Piloting

The low-carbon city piloting (LCC) is defined as follows: if the registered city of a listed enterprise implements low-carbon piloting, LCC = 1 in the current and following years; otherwise, LCC = 0. During the sample period, two batches of pilot cities were announced. Hence, the first and second batches of pilot cities were selected as the treatment group. Some cities belong to both batches. As a result, the start time of piloting of a province was taken as that of every city administered by that province.

#### 3.3.2. EIE Measurement

The EIE was measured mainly referring to the research of Biddle et al. [27] and Choi et al. [28]. Using the enterprise expected investment model of Richardson [29], this paper first calculates the normal investment level expected by the enterprise and then measures the EIE with the regression residual of the model.

The model can be expressed as follows:

(2) $$\begin{array}{c} {\text{Inv}}_{i,t}=\beta_{0}+\beta_{1}{\text{Growth}}_{i,t-1}+\beta_{2}{\text{Lev}}_{i,t-1}+\beta_{3}{\text{Age}}_{i,t-1}+\beta_{4}{\text{Size}}_{i,t-1}+\beta_{5}{\text{Cash}}_{i,t-1}+\beta_{6}{\text{Ret}}_{i,t-1}+\beta_{7}{\text{Inv}}_{i,t-1}+\sum \text{Y}\text{ear}+\sum \text{I}\text{ndustry}+\varepsilon_{i,t}, \end{array}$$

where Inv_*i*,*t*_ is the investment level of the enterprise in year *t*, which is measured by the ratio of the cash paid for the purchase and construction of fixed assets, intangible assets, and other long-term investments to the total assets at the beginning of the period, and Growth_*i*,*t*−1_, Lev_*i*,*t*−1_, Age_*i*,*t*−1_, Size_*i*,*t*−1_, Cash_*i*,*t*−1_, Ret_*i*,*t*−1_, and Inv_*i*,*t*−1_ are the growth capacity, debt rate, listing period, company scale, cash holding ratio, stock return, and investment level of the enterprise in year *t* − 1, respectively.

The regression residual *ε*_*i*,*t*_ reflects the inefficient investment expenditure of the enterprise. If *ε*_*i*,*t*_ > 0, then the investment is excessive; if *ε*_*i*,*t*_ < 0, then the investment is insufficient. The absolute value of the residual *ε*_*i*,*t*_ was taken to measure the EIE (Investeff). This value reflects how much the enterprise investment deviates from the theoretical expectation. The greater the value, the larger the deviation and the lower the EIE.

### 3.4. Control Variables and Measurement

The HDID model controls the key explanatory variables and solves the endogeneity induced by the correlation between time-invariable individual features. But the time-varying individual features should be controlled to reduce the estimation inconsistency arising from missing variables. Referring to the literature, this paper selects the following control variables: enterprise size (Size), price-earnings ratio (PE), government subsidy change (Subchange), holding concurrent positions of chairman and general manager (Dual), industry concentration (Hhi), and sustainable growth rate (Sgr). In addition, industrial and provincial dummy variables were included. Reasons for choosing the control variables are as follows: firstly, the existing research has shown that enterprises of different scales have different financing constraints, which affect EIE differently. Secondly, *price-earnings ratio* has been used as a key variable to measure investor sentiment, which has been proved to bear on the investment behavior of enterprises through equity financing, catering, manager optimism, debt financing, and other channels. Thirdly, the local government would intervene in the economic operation of enterprises by means of government subsidies, guiding local investment, and changing the investment direction and level of enterprises. Fourthly, the duality of chairman and general manager, as an important allocation mechanism of decision-making power, directly affects EIE. Fifthly, market competition can improve information sharing. In a fully competitive market, owners will have reliable information of managers. Thus, the information asymmetry between shareholders and management is mitigated, so that executives will not expand blindly or get complacent, and the enterprises will invest more efficiently. Sixthly, the sustainable growth rate reflects the sustainability of enterprises. The sustainable growth rate can affect EIE through earnings retention and financial structure.

## 4. Empirical Results and Analysis

### 4.1. Benchmark Regression

Table 1 lists the regression results of LCCP on EIE. The results show that the regression coefficient of LCCP on EIE is significantly negative, regardless of whether the time fixed effect, industry fixed effect, provincial fixed effect, and control variables are controlled. Since *Investeff* represents the deviation of enterprise investment from the theoretical expectation, the greater the deviation, the lower the EIE. Hence, the empirical results reveal that LCCP significantly enhances EIE. According to column (5) of Table 1, after controlling time fixed effect, industry fixed effect, provincial fixed effect, and control variables in the model, the regression coefficient of LCCP on EIE was -0.005 (significant at the level of 5%), which indicates that the EIE in low-carbon city pilot areas is 0.5% higher than that of enterprises in non-low-carbon city pilot areas. Hypothesis 1 was therefore validated.

Next, EIE was divided into excessive investment and insufficient investment and treated as the explained variable separately. On this basis, model (1) was regressed again. The empirical results are shown in Table 2. It can be seen that LCCP mainly affects EIE by solving the insufficient investment, without easing excessive investment.

### 4.2. Parallel Trend Testing

Parallel trends are the premise of DID. In view of the relevant studies, this paper adopts event-based analytics to test the parallel trends [30, 31]. The model can be expressed as

(3) $$\begin{array}{c} \text{Investef}f_{i,t+1}=\alpha +\overset{6}{\underset{k\geq -5}{\sum }}\beta_{k}D_{i,t}^{k}+{X_{i,t}}^{\prime }\gamma +\mu_{i}+\sum \text{Y}\text{ear}+\sum \text{I}\text{ndustry}+\sum \text{P}\text{rovince}+\varepsilon_{i,t}, \end{array}$$

where Investeff is EIE; *D*^*k*^_*i*,*t*_ is a series of dummy variables, indicating the *k*-th year since the implementation of low-carbon city piloting (*k* ∈ [−5, 6] and *k* ≠ 0). This paper mainly considers parameter *β*_*k*_ (*k* ∈ [−5, −1]). The other variables in formula (3) are configured consistently as those in benchmark model (1). If *k* < 0 and if *β*_*k*_ is not significantly different from zero, then parallel trends are satisfied.

Figure 1 reports the estimated value of *β*_*k*_ and the confidence interval of 95%. It can be seen that when *k* < 0, the null hypothesis that estimated value of *β*_*k*_ is zero cannot be rejected. This mean, before low-carbon city piloting, the treatment group and the control group meet the parallel trend hypothesis after the relevant variables are controlled.

### 4.3. Robustness Tests

The following robustness tests were carried out.

#### 4.3.1. Nonrandom Selection of Samples

The first batch of low-carbon pilot cities in China was designated by the superior government. As for the second and third batches, application and expert review were added as necessary links of determining low-carbon pilot cities. Thus, the list of low-carbon pilot cities is not determined purely by random. To mitigate the negative effect of nonrandom selection on estimation results, this paper adds the cross-term Sc · *f*(*t*) between city attribute and time trend to the benchmark regression model, where Sc is the city attribute (whether the city is the provincial seat or a special economic zone) and *f*(*t*) is the first-order term of the time trend. The cross-term controls the time-varying influence of the intrinsic difference between city attributes over EIE. The regression results are recorded in column (1) of Table 3.

#### 4.3.2. Placebo Test

The approval time of low-carbon pilot cities was moved ahead by 3 years, and variable Before_3 was added to model (1). The regression results are displayed in columns (2) and (3) of Table 3. It can be seen that the variable did not significantly affect excessive or insufficient investment.

#### 4.3.3. Abnormal Value Removal

Considering the effect of its abnormal value, the explained variable was censored at the 1% and 99% quantiles. The regression results are displayed in column (4) of Table 3.

#### 4.3.4. Controlling the Influence of the Level of Economic Development in the Registered City on EIE

Per capita gross domestic product (GDP) was added to the benchmark model. The regression results are shown in column (5) of Table 3.

#### 4.3.5. Influence of the Other Policies

Two cross-terms were designed: the cross-term between whether the city is a new energy demonstration city and the time of approval (Ncity) and the cross-term between the city environmental protection criticized by superiors and the time of criticized (HBYT). The two terms were introduced to model (1). The regression results are given in columns (6) and (7) of Table 3.

#### 4.3.6. Removal of Provinces without Pilot Cities

To increase the similarity between treatment group and control group, this paper further removes the provinces without any pilot cities. The regression results are displayed in column (8) of Table 3. After a series of robustness tests, the main conclusions of this paper still hold.

## 5. Heterogeneity Analysis

### 5.1. Urban Green Culture

Regarding the measurement of urban green culture, this paper selects the actual year-end number public vehicles and trams/(the actual year-end number public vehicles and trams+the actual year-end number of taxis) to depict the green consumption concept of residents. The samples were grouped by the median of the variable and tested separately. The results are shown in columns (1) and (2) of Table 4. The results show that, in areas with strong green culture, LCCP has a positive effect on EIE. Hypothesis 6 is thereby testified.

To rule out the possibility that the above results are caused by government intervention, this paper uses the government-market relationship index compiled by Fan et al. [32] to measure the degree of intervention of Chinese local governments and divides the samples into high intervention group and low intervention group by the median of the variable. The regression results are shown in columns (3) and (4) of Table 4. It can be seen that the effect of LCCP on EIE is significantly negative in the low intervention areas, but not significant in the high intervention areas. The impact of government intervention is thus excluded.

Compared with non-resource-based cities, many resource-based cities in China lag behind in the construction of urban green culture, due to their long-term dependence on resources. According to the *National Sustainable Development Plan for Resource-Based Cities (2013-2020)*, this paper divides cities into resource-based cities and non-resource-based cities and performs regression on each group. The results are shown in columns (5) and (6) of Table 4. It is found that, in resource-based cities, low-carbon pilot policies have no significant impact on EIE, while in non-resource-based cities, these policies have a significant positive impact on EIE. This further demonstrates the positive role of urban green culture.

### 5.2. Urban Confucian Culture

Referring to the research of Du [33], this paper selects the distance between the enterprise's registered place and the seven existing Confucian cultural centers in China to measure the influence of Confucian culture. These centers were gradually formed by the spread of Confucianism in China for more than 2,500 years, including Qilu in Shandong, Chengdu in Sichuan, Luoyang in Henan, Sanming and Longyan in Fujian, Dongtai in Jiangsu, and Ningbo and Shaoxing in Zhejiang. Referring to Baidu Map, the authors collected the longitude and latitude coordinates of the above seven Confucian centers, as well as the longitude and latitude coordinates of the registration places of all A-share listed companies. These data were used to calculate the mean distance between the registration places of each listed company and each Confucian center. The larger the value of Confucian culture (Confu), the higher the degree of influence of Confucian culture on the enterprise. The samples were grouped by the median of Confu and divided into a weak Confucian culture group and a strong Confucian culture group. The two groups were regressed separately, and the results are shown in Table 5. It was found that in weak Confucian culture areas, LCCP has no significant effect on EIE, while in strong Confucian culture areas, LCCP significantly improves EIE. Hypothesis 7 is therefore verified.

### 5.3. Industrial Heterogeneity of Carbon Emissions

Under the influence of green culture and Confucian culture, enterprises identify with different goals and pursue legitimacy to different degrees. This paper holds that LCCP has a more positive impact on the EIE in high-carbon emission industries than low-carbon emission industries. To test this hypothesis, the industries were divided into high-emission industry, medium-emission industry, and low-emission industry, according to the trisectional quantiles of carbon emissions of all industries in China, in reference of the carbon emission data in 2009. The relevant data come from Carbon Emission Accounts & Datasets (CEADs). The regression results are shown in Table 6. It was learned that, compared with that in low-emission industries, LCCP has a significant positive impact on the EIE in high-emission industries. This is in line with the original policy intention of low-carbon city piloting. To improve the robustness of the results, this paper combines the medium-emission group and the low-emission group before starting a new robustness test. The regression results are still consistent.

## 6. Influence Mechanism Analysis

The impact of LCCP on EIE mainly manifests as three effects, namely, technological innovation effect, financing constraint effect, and resource allocation effect. These effects are tested separately in this paper.

### 6.1. Technological Innovation Effect

The R&D expenditure reflects the willingness of enterprises to invest in technological innovation. Therefore, this paper selects R&D expenditure as a proxy variable for technological innovation and measures the variables with the ratio of R&D expenditure to operating income. The regression results are shown in column (1) of Table 7. It can be seen that LCCP boosts the R&D expenditure of enterprises, indicating that LCCP enhances EIE through the effect of technological innovation. Hypothesis 3 is therefore verified.

### 6.2. Financing Constraint Effect

Scholars mainly use KZ, WW, and SA indices to measure the financing constraint of enterprises [34, 35]. Among them, KZ is the most widely used measure, owing to the maturity of its theories. Drawing on Kaplan and Zingales' methodologies, this paper constructs the KZ index to measure the financing constraint of enterprises. The regression results are shown in column (2) of Table 7. It can be seen that LCCP can effectively alleviate the financing constraint of enterprises; i.e., LCCP promotes EIE by alleviating enterprise financing constraint. Hypothesis 4 is thereby validated.

### 6.3. Resource Allocation Effect

This paper uses capital allocation efficiency as a proxy variable of resource allocation efficiency and designs model (4) following the investment-investment opportunity sensitivity model:

(4) $$\begin{array}{c} {\text{invest}}_{i,t}=\partial_{0}+\partial_{1}{\text{LCC}}_{i,t}\times {\text{ROA}}_{i,t}+\partial_{2}{\text{LCC}}_{i,t}+\partial_{3}{\text{ROA}}_{i,t}+{X_{i,t}}^{\prime }\gamma +\mu_{i}+\sum \text{Y}\text{ear}+\sum \text{I}\text{ndustry}+\sum \text{P}\text{rovince}+\varepsilon_{i,t}, \end{array}$$

where invest is the investment level of the enterprise, which is equal to (cash paid for the purchase and construction of fixed assets, intangible assets, and other long − term assets − cash recovered from the disposal of fixed assets, intangible assets, and other long − term assets)/total year − end assets, and ROA is the return on assets used to measure enterprise investment opportunities; the coefficient of the cross-term between LCC and ROA measures the impact of LCCP on the efficiency of enterprise resource allocation; the definitions of other variables are consistent with model (1). The regression results are shown in column (3) of Table 7. It can be seen that LCCP does not significantly improve the resource allocation efficiency of enterprises. Hypothesis 5 is therefore falsified.

## 7. Conclusions and Policy Implications

This paper measures the EIE with the Richardson enterprise expectation investment model. The research samples are the A-share listed nonfinancial enterprises in Shanghai and Shenzhen stock exchanges of China from 2007 to 2016. On this basis, the impact of LCCP on EIE was estimated by using HTDID, and the heterogeneous effect of urban culture was also investigated.

The main conclusions are as follows:

(1) Overall, LCCP improves EIE, and the research conclusion passes a series of robustness tests. (2) Mechanism analysis reveals that LCCP mainly acts on EIE along two paths: promoting enterprise technological innovation and easing financing constraint. But the LCCP does not have a significant effect on resource allocation. (3) The influence of LCCP over EIE varies with urban cultures. The ecological wisdoms of green urban culture and Confucian culture, such as benevolence to all beings and the harmony between man and nature, help to enhance the promoting effect of LCCP on EIE

The policy implications are as follows:

First, the positive effect of LCCP on EIE was demonstrated through empirical research. The construction of low-carbon cities is an important means for European developed countries to improve residents' well-being and urban competitiveness. In developing countries, the legal system is relatively weak, and the relevant pilot policies may be difficult to implement. The research results prove that LCCP has the same ideal effect in developing countries like China and can be used as an important means to promote high-quality economic development.

Second, strengthening urban cultural governance is of great significance to LCCP promotion. Urban cultural governance focuses on improving the cultural connotation and quality of urban governance. This is particularly true as China witnesses increasing urban scale, rapid construction, the lack of urban culture, and cultural imbalances. Then, it is necessary to highlight the construction of cultural soft power in governance goals and contents. Special attention should be paid to urban cultural governance from the perspective of green development, making cultural governance a powerful guarantee for promoting the progress of urban civilization and green development.

## Figures and Tables

**Figure 1:** DID parallel trend testing results.

**Table 1:** Benchmark regression results.

Variables	(1)	(2)	(3)	(4)	(5)
	HTDID	HTDID	HTDID	HTDID	HTDID
LCC	-0.004^∗∗∗^	-0.004^∗∗^	-0.008^∗∗∗^	-0.008^∗∗∗^	-0.005^∗∗^
	(-2.60)	(-2.30)	(-4.04)	(-3.91)	(-2.25)

Size					-0.008^∗∗∗^
					(-3.74)

PE					0.000
					(1.23)

Subchange					0.008
					(1.34)

Dual					0.008^∗∗^
					(2.27)

Hhi					0.061
					(1.15)

Sgr					0.010
					(1.48)

Constant	0.046^∗∗∗^	-0.007	0.047^∗∗∗^	-0.040	0.026
	(8.04)	(-0.29)	(26.44)	(-1.34)	(0.64)

Observations	18,569	18,604	14,846	14,823	10,951

*R*-squared	0.004	0.009	0.001	0.017	0.024

Control variables	No	No	No	No	Yes

Time fixed effects	No	No	Yes	Yes	Yes

Enterprise fixed effects	Yes	Yes	Yes	Yes	Yes

Province fixed effects	No	Yes	No	Yes	Yes

Industry fixed effects	Yes	No	No	Yes	Yes

Note: robust *t*-statistics are in parentheses; ^∗∗∗^*p* < 0.01, ^∗∗^*p* < 0.05, and ^∗^*p* < 0.1.

**Table 2:** Influence of LCCP on excessive and insufficient EIEs.

Variables	(1)	(2)
	Excessive investment	Insufficient investment
LCC	-0.006	-0.005^∗∗∗^
	(-0.88)	(-3.30)

Constant	0.154^∗^	-0.005
	(1.85)	(-0.22)

Observations	3,900	7,051

*R*-squared	0.054	0.036

Control variables	Yes	Yes

Time fixed effects	Yes	Yes

Enterprise fixed effects	Yes	Yes

Province fixed effects	Yes	Yes

Industry fixed effects	Yes	Yes

Note: robust *t*-statistics are in parentheses; ^∗∗∗^*p* < 0.01, ^∗∗^*p* < 0.05, and ^∗^*p* < 0.1.

**Table 3:** Regression results of robustness tests.

Variables	(1)	(2)	(3)	(4)	(5)	(6)	(7)	(8)
	Nonrandom selection of samples	Placebo test	Placebo test	Abnormal value removal	Controlling level of economic development	New energy demonstration city	Environmental criticism	Removal of provinces without pilot cities
LCC	-0.005^∗∗^			-0.005^∗∗^	-0.005^∗∗^	-0.007^∗∗∗^	-0.005^∗∗^	-0.006^∗∗^
	(-2.32)			(-2.36)	(-2.30)	(-2.80)	(-2.31)	(-2.40)

Before_3		-0.020	-0.004					
		(-1.17)	(-1.55)					

PGDP					0.000			
					(0.59)			

Ncity						0.002		
						(0.60)		

HBYT							-0.007^∗^	
							(-1.75)	

Constant	0.027	0.168^∗^	-0.001	0.016	0.024	0.041	0.026	0.010
	(0.66)	(1.88)	(-0.02)	(0.43)	(0.58)	(1.02)	(0.64)	(0.22)

Observations	10,951	3,900	7,051	10,951	10,894	9,724	10,951	9,840

*R*-squared	0.024	0.054	0.034	0.023	0.024	0.020	0.024	0.023

Sc · *f*(*t*)	Yes							

Control variables	Yes	Yes	Yes	Yes	Yes	Yes	Yes	Yes

Time fixed effects	Yes	Yes	Yes	Yes	Yes	Yes	Yes	Yes

Enterprise fixed effects	Yes	Yes	Yes	Yes	Yes	Yes	Yes	Yes

Province fixed effects	Yes	Yes	Yes	Yes	Yes	Yes	Yes	Yes

Industry fixed effects	Yes	Yes	Yes	Yes	Yes	Yes	Yes	Yes

Note: robust *t*-statistics are in parentheses; ^∗∗∗^*p* < 0.01, ^∗∗^*p* < 0.05, and ^∗^*p* < 0.1.

**Table 4:** Regression results of green culture heterogeneity.

Variables	(1)	(2)	(3)	(4)	(5)	(6)
	Strong green culture	Weak green culture	High intervention	Low intervention	Resource-based city	Non-resource-based city
LCC	-0.011^∗∗^	-0.007^∗^	-0.003	-0.007^∗∗^	-0.005	-0.006^∗∗^
	(-2.53)	(-1.73)	(-0.69)	(-2.35)	(-0.46)	(-2.29)

Constant	0.054	0.061	0.058	-0.044	0.040	0.044
	(1.31)	(1.49)	(1.38)	(-1.42)	(0.84)	(1.10)

Observations	4,896	4,498	4,792	6,116	1,109	9,842

*R*-squared	0.014	0.067	0.041	0.016	0.032	0.025

Control variables	Yes	Yes	Yes	Yes	Yes	Yes

Time fixed effects	Yes	Yes	Yes	Yes	Yes	Yes

Enterprise fixed effects	Yes	Yes	Yes	Yes	Yes	Yes

Province fixed effects	Yes	Yes	Yes	Yes	Yes	Yes

Industry fixed effects	Yes	Yes	Yes	Yes	Yes	Yes

Note: robust *t*-statistics are in parentheses; ^∗∗∗^*p* < 0.01, ^∗∗^*p* < 0.05, and ^∗^*p* < 0.1.

**Table 5:** Regression results of Confucian culture heterogeneity.

Variables	(1)	(2)
	Weak Confucian culture	Strong Confucian culture
LCC	-0.004	-0.008^∗∗^
	(-1.07)	(-2.41)

Constant	0.030	0.016
	(0.64)	(0.37)

Observations	5,194	5,757

*R*-squared	0.035	0.023

Control variables	Yes	Yes

Time fixed effects	Yes	Yes

Enterprise fixed effects	Yes	Yes

Province fixed effects	Yes	Yes

Industry fixed effects	Yes	Yes

Note: robust *t*-statistics are in parentheses; ^∗∗∗^*p* < 0.01, ^∗∗^*p* < 0.05, and ^∗^*p* < 0.1.

**Table 6:** Regression results of industrial heterogeneity in carbon emissions.

Variables	(1)	(2)	(3)	(4)
	High emissions	Median emissions	Low emissions	Medium- and low-emission industries
LCC	-0.009^∗^	-0.000	-0.003	-0.003
	(-1.81)	(-0.11)	(-0.49)	(-1.05)

Constant	0.078^∗^	0.009	0.220^∗∗∗^	0.113
	(1.78)	(0.23)	(2.83)	(1.60)

Observations	3,974	3,483	2,910	6,393

*R*-squared	0.033	0.045	0.048	0.033

Control variables	Yes	Yes	Yes	YES

Time fixed effects	Yes	Yes	Yes	YES

Enterprise fixed effects	Yes	Yes	Yes	YES

Province fixed effects	Yes	Yes	Yes	YES

Industry fixed effects	Yes	Yes	Yes	YES

Note: robust *t*-statistics are in parentheses; ^∗∗∗^*p* < 0.01, ^∗∗^*p* < 0.05, and ^∗^*p* < 0.1.

**Table 7:** Regression results of influence mechanisms.

Variables	(1)	(2)	(3)
	Technological innovation effect	Financing constraint effect	Resource allocation effect
LCC∗ROA			-0.043
			(-0.91)

LCC	0.007^∗∗∗^	-0.115^∗∗^	0.009^∗∗∗^
	(3.63)	(-2.11)	(3.01)

ROA			0.065^∗∗^
			(2.34)

Constant	0.039^∗∗∗^	-0.966	-0.010
	(3.06)	(-0.87)	(-0.37)

Observations	10,158	15,071	13,198

*R*-squared	0.182	0.228	0.093

Control variables	Yes	Yes	Yes

Time fixed effects	Yes	Yes	Yes

Enterprise fixed effects	Yes	Yes	Yes

Province fixed effects	Yes	Yes	Yes

Industry fixed effects	Yes	Yes	Yes

Note: robust *t*-statistics are in parentheses; ^∗∗∗^*p* < 0.01, ^∗∗^*p* < 0.05, and ^∗^*p* < 0.1.

## Data Availability

The data used to support the findings of this study are available from the corresponding author upon request.
